The article "AEG-1/miR-221 Axis Cooperatively Regulates the Progression of Hepatocellular Carcinoma by Targeting PTEN/PI3K/AKT Signaling Pathway" was retracted in 2022. Reasons: manipulated images; duplicated images; unreliable results or conclusions.

# AEG-1/miR-221 Axis Cooperatively Regulates the Progression of Hepatocellular Carcinoma by Targeting PTEN/PI3K/AKT Signaling Pathway

**DOI:** 10.3390/ijms20225526

**Published:** 2019-11-06

**Authors:** Maheshkumar Kannan, Sridharan Jayamohan, Rajesh Kannan Moorthy, Siva Chander Chabattula, Mathan Ganeshan, Antony Joseph Velanganni Arockiam

**Affiliations:** 1 Molecular Oncology Laboratory, Department of Biochemistry, School of Life Sciences, Bharathidasan University, Tiruchirappalli 620024, India; kmaheshkumar02@gmail.com (M.K.); sridharan2011phd@gmail.com (S.J.); adsrajeshkannan1987@gmail.com (R.K.M.); 2 Department of Biotechnology, Bhupat and Jyoti Mehta School of Biosciences, Indian Institute of Technology Madras, Chennai 600036, India; siva.chabathula@gmail.com; 3 Cancer Biology Laboratory, Department of Biomedical Science, School of Life Sciences, Bharathidasan University, Tiruchirappalli 620024, India; mathan@bdu.ac.in

**Keywords:** miR-221, astrocyte elevated gene-1, HCC, cell proliferation, regulatory proteins

## Abstract

Hepatocellular carcinoma (HCC) is the third leading malignancy worldwide, causing mortality in children and adults. AEG-1 is functioned as a scaffold protein for the proper assembly of RNA-induced silencing complex (RISC) to optimize or increase its activity. The increased activity of oncogenic miRNAs leads to the degradation of target tumor suppressor genes. miR-221 is an oncogenic miRNA, that plays a seminal role in carcinogenesis regulation of HCC. However, the molecular mechanism and biological functions of the miR-221/AEG-1 axis have not been investigated extensively in HCC. Here, the expression of miR-221/AEG-1 and their target/associate genes was analyzed by qRT-PCR and Western blot. The role of the miR-221/AEG-1 axis in HCC was evaluated by proliferation assay, migration assay, invasion assay, and flow cytometry analysis. The expression level of miR-221 decreased in AEG-1 siRNA transfected HCC cells. On the other hand, there were no significant expression changes of AEG-1 in miR-221 mimic and miR-221 inhibitor transfected HCC cells and inhibition of miR-221/AEG-1 axis decreased cell proliferation, invasion, migration, and angiogenesis and induced apoptosis, cell cycle arrest by upregulating p57, p53, PTEN, and RB and downregulating LSF, MMP9, OPN, Bcl-2, PI3K, AKT, and LC3A in HCC cells. Furthermore, these findings suggest that the miR-221/AEG-1 axis plays a seminal oncogenic role by modulating PTEN/PI3K/AKT signaling pathway in HCC. In conclusion, the miR-221/AEG-1 axis may serve as a potential target for therapeutics, diagnostics, and prognostics of HCC.

## 1. Introduction

Hepatocellular carcinoma (HCC) is the fifth common malignancy and observed third leading cancer-caused death with a limited prediction [1]. HCC is the highest incidence and most rising cancer following others in developing countries like India [2]. Hepatitis B virus (HBV) and hepatitis C virus (HCV) are the major risk factor for human HCC. Most of HCC patients suffer from HBV infections, approximately 50–80% of cases, and 10 to 25% of HCV [3]. Non-alcoholic fatty liver disease (NAFLD) is another important disease caused by the accumulation of fat exceeding 5% of liver weight in the absence of alcohol. NAFLD is the major cause of liver damage that leads to liver cirrhosis and HCC [4]. NAFLD is the major non-viral risk factor for developing HCC worldwide. In India, 9–32% of cases affected by NAFLD are associated with HCC [5]. Surgery is considered as the primary treatment for HCC. Recent studies showed that chemotherapy is the best treatment for HCC [6]. However, the overall survival time of drug-treated patients is only up to two to five years [7]. A better approach to improve the molecular biological studies and targeted therapy for the regulatory networks of cell proliferation, apoptosis, and angiogenesis progression could be more effective in the treatment of HCC.

MicroRNAs (miRNAs) are a class of short endogenous noncoding RNAs (18–25 nucleotides in length), and it acts as oncogenes or tumor suppressors that dysregulate target gene expression at the post-transcription level [8,9]. It is considered as a key mediator in the various biological processes, including differentiation, proliferation, apoptosis, and angiogenesis via degradation of specific target mRNA [10,11] or signaling pathways, such as PTEN/PI3K/AKT [12] signaling targeted by several miRNAs, especially miR-221/222 [13], miR-181a/b-1 [14], miR-146b [15], and miR-543 [16] through binding at their 3′ UTR (untranslated region). Besides, miRNAs are involved in the progression of NAFLD in different cell types and considered as some of the potential biomarkers [4]. Increasing evidence suggests that both oncogenic or tumor suppressor miRNAs are associated with many human diseases and play an acquired role in cancer initiation, progression especially, miR-221 acts as an oncogene and induces malignant activities in human cancers, including HCC [17,18,19], but the specificity and sensitivity of miR-221 have been explored to a certain extent in HCC.

Astrocyte elevated gene-1 (AEG-1) called Metadherin (MTDH) or LYRIC is reported as human immunodeficiency virus (HIV)-1 and tumor necrosis factor-a (TNF-a)-inducible gene in human fetal astrocytes [20,21]. AEG-1 is frequently overexpressed in multiple human malignancies, including HCC. However, the clinical studies on AEG-1-mediated tumor progression are still inconclusive. AEG-1 plays several crucial roles in promoting cancer development, tumor progression, through the development of invasion, migration, evasion of apoptosis, angiogenesis, and chemoresistance. In addition to that, ectopic expression of AEG-1 converts non-tumorigenic into highly aggressive tumors by dysregulating specific regulatory genes and signaling pathways, especially PI3K/AKT [22,23]. AEG-1 is functioned as a scaffold protein for the proper assembly of the RISC complex and increases the activity of oncogenic miRNA. The increased activity of oncogenic miRNA leads to the degradation of target genes [24].

Recent studies showed miR-221 is overexpressed and regulated as an individual or cluster in HCC [25,26]. On the other hand, AEG-1 is regulated by multiple miRNAs during carcinogenesis of HCC [25,27]. Moreover, few studies have investigated the regulative network axis, particularly miR-221 target genes (PHF2 [25], C1QTNF1-AS1 [26], and miRNAs (miR-375 [27,28] and miR-195 [29]) targeting AEG-1 in HCC. Since the studies on the miR-221/AEG-1 axis on target/associate genes in HCC are still limited and unclear, we aimed to analyze the molecular mechanism of the miR-221/AEG-1 axis and possible targets in HCC.

## 2. Results

### 2.1. miR-221/AEG-1 Overexpressed in HCC Cell Lines

We examined the expression of miR-221 and AEG-1 in three HCC cell lines (HepG2, Huh7, and Hep3B) and THLE-2 by qRT-PCR. The results showed that the expression of miR-221 and AEG-1 was significantly increased in all HCC cell lines when compared to THLE-2 (Figure 1A,B). Next, we examined miR-221 expression in miR-221 mimic (Figure 1C), miR-221 inhibitor (Figure 1D), and AEG-1 siRNA (Figure 1E) transfected HCC cells. miR-221 expression decreased in miR-221 inhibitor and AEG-1 siRNA transfected group and increased in miR-221 mimic transfected group. Subsequently, we analyzed the AEG-1 expression in miR-221 mimic, miR-221 inhibitor, and AEG-1 siRNA transfected group. AEG-1 expression does not change in miR-221 mimic, and miR-221 inhibitor transfected cells (Figure 1F) and decreased in AEG-1 siRNA transfected HCC cells (Figure 1G).

### 2.2. miR-221/AEG-1 Axis Regulates Apoptosis, Cell Cycle, Angiogenesis and Autophagy Mechanism by the Activation of Regulatory Genes in HCC Cells In Vitro

We examined the effect of miR-221/AEG-1 on cell regulatory mRNA expression level by transfecting miR-221 mimic, miR-221 Inhibitor, AEG-1 siRNA, and their negative controls in HCC cells by qRT-PCR. The regulative mRNA expressions of angiogenesis (LSF and MMP9), anti-apoptotic (OPN, and Bcl2), autophagy (LC3A) and PI3K/Akt were decreased and cell cycle regulatory mRNA expressions (PTEN, p57, p53, and RB) were increased (Figure 2 and Figure 3) in miR-221 inhibitor and AEG-1 siRNA transfected HCC cells. The results showed that miR-221 and AEG-1 could play an important role in regulatory networks of HCC.

### 2.3. Knockdown of miR-221 and AEG-1 Inhibits Cellular Proliferation, Migration, Invasion and Tube Formation In Vitro

To investigate the role of AEG-1 and miR-221 in cell migration, invasion, and angiogenesis we used wound healing, transwell, and tube formation assay performed in miR-221 mimic, miR-221 inhibitor, AEG-1 siRNA and their controls transfected HCC and HUVECs cells in in vitro. As presented in Figure 4A–C, wound healing assay confirmed that miR-221 inhibitor and AEG-1 siRNA effectively suppressed the cell migration in HCC cells when compared to their control. Furthermore, miR-221 and AEG-1 effectively inhibited the cell proliferation in HCC cells (Figure 4D), which was confirmed by MTT assay. Moreover, transwell assay indicated that the downregulation of miR-221 and AEG-1 effectively inhibits cell invasiveness (Figure 5A) and migration (Figure 5B) compared to the corresponding controls and miR-221 mimic transfected HCC cells.

Next, we performed a capillary-like tube formation assay to analyze the effect of AEG-1 and miR-221 in tumor angiogenesis. As shown in Figure 5C, tube networks are poorly connected and reduce the tube formation in miR-221 inhibitor and AEG-1 siRNA transfected HUVEC cells compared to control. From these results, we identified miR-221 and AEG-1 as a potential angiogenesis regulator in HUVEC cells.

### 2.4. Downregulation of miR-221 and AEG-1 Promotes Apoptosis and Cell Cycle Arrest in HCC Cells In Vitro

To further confirm the regulation of miR-221 and AEG-1 in HCC cell cycle and apoptosis by flow cytometry. HCC cells transfected with mock control, inhibitor negative control, miR-221 mimic, miR-221 inhibitor, and AEG-1 siRNA and cell cycle analysis was performed using PI staining and apoptosis measured using Annexin V-FITC/PI duel-staining with Alexa Fluor-conjugation. Knockdown of miR-221 and AEG-1 in HepG2, Huh7, and Hep3B cells showed the percentage of peaks in G0/G1 (Figure 6A), sub-G1, and G2/M phase (Figure 6B) increased compared to controls. Meanwhile, there were no changes in cell cycle and apoptotic level in miR-221 mimic transfected HCC cells compared to control. As Figure 6A, B shows, miR-221/AEG-1 axis could be majorly involved in and regulate the HCC cell cycle and cell death.

### 2.5. Downregulation of miR-221 and AEG-1 Inhibits Angiogenesis, and Enhance Apoptosis, Cell Cycle Arrest by Modulating Regulatory Proteins In Vitro

We observed the relative protein expression of AEG-1 in HepG2, Huh 7, Hep3B, and THLE-2 cells (Figure 7A). Next, we analyzed the relative AEG-1 expression in miR-221 mimic, miR-221 inhibitor, AEG-1 siRNA and their controls transfected HCC cells. AEG-1 protein expression level did not alter in miR-221 mimic, miR-221 inhibitor and their corresponding control transfected HCC cells, and decreased in AEG-1 siRNA transfected HCC cells when compared to their controls. (Figure 7B). Additionally, we evaluated the effect of miR-221 and AEG-1 inhibition on cellular regulatory proteins. Knockdown of miR-221 and AEG-1 downregulates LSF, MMP9, and upregulates p57, p53, and RB protein levels in HepG2 (Figure 7C), Huh7 (Figure 7D), and Hep3B (Figure 7E) cells. Moreover, knockdown of miR-221 and AEG-1 upregulates PTEN and downregulates OPN, Bcl-2, LC3A/B and PI3K/p-Akt protein levels in HepG2 (Figure 8A), Huh7 (Figure 8B), and Hep3B (Figure 8C) cells. However, expression of these proteins deregulated in miR-221 mimic transfected HCC cells compared to controls. Therefore, miR-221 and AEG-1 have been identified as the potential oncogenes in HCC.

## 3. Discussion

In recent years, cancer has been one of the most challenging issues in global healthcare. Cancer treatment, such as chemotherapy has significantly improved the overall patient survival. Nevertheless, the ability of cancer prevention and early diagnosis are still a challenge. Cancer is the only disease which affects healthy cells without injury. Nowadays, the identification and targeting the tumor antigens are considered as the advanced treatment for cancer [30]. HCC is the most rising cancer following others in developing countries like India. HBV is the major risk factor for HCC [31], and it promotes cell proliferation by targeting oncogenes and onco-miRNAs, especially miR-221 [32] and AEG-1 [33].

Tumor-associated antigen (TAA) is one of the tumor antigens overexpressed in tumor cells. Earlier studies identified 15 targets of TAA, and characterized namely astrocyte elevated genes. AEG-1 is one of the 15 targets identified in vivo and TAA is also assumed to be a component of RNA-induced silencing complex (RISC), which is involved in miRNA interactions [20,21,34]. It plays a crucial role in tumorigenesis by over expressing and regulating metastasis, chemoresistance, migration, and apoptosis in HCC [28]. These studies strongly represent that AEG-1 is a frequently overexpressed oncogene and is correlated to several hallmarks of human HCC. We found that AEG-1 was significantly upregulated in HCC cells, which indicated its potential therapeutic target for liver carcinogenesis.

Accumulating evidence shows that miRNAs contributes to many human pathological processes, including cancer, and acts as a tumor suppressor or oncogene, and regulates cell differentiation, apoptosis, chemoresistance, proliferation, survival, metastasis, and malignant activities by the activation or suppression of target mRNAs in different types of cancers, including HCC [13,14]. Most of the cancer studies show that miR-221 is significantly overexpressed and regulates all the above-mentioned process. This evidence revealed that miR-221 might play a vital role in human carcinogenesis, including HCC [17,18,19]. We showed the ectopic expression of miR-221 that indicates the tumorigenic function of miR-221 in HCC. Previous studies reported that AEG-1 is a direct target of tumor suppressor miRNAs miR-375 and miR-195 confirmed by luciferase reporter assay and downregulated the expression of these miRNAs during carcinogenesis. The overexpression of tumor suppressor miRNAs inhibits cellular proliferation, invasion, migration, metastasis, and angiogenesis by the downregulation of AEG-1 in HCC [8,27,28,29] and cervical cancer cells [11]. On the other hand, overexpression of miR-221 promotes cell proliferation, metastasis by the dysregulation of tumor suppressors and oncogenes in HCC [24,25,26]. Moreover, miR-221 regulates angiogenesis and knockdown of miR-221 inhibits SND1-mediated angiogenesis activity in HCC cells [35].

This result demonstrates that miR-221 and AEG-1 have an oncogenic role and majorly regulate human carcinogenesis. Downregulation of miR-221 and AEG-1 inhibits cell differentiation, metastasis, invasion, migration, and angiogenesis in human cancers, including HCC. Thus, we concluded that the downregulation of both miRNA-221 and AEG-1 inhibits the activity of cell proliferation, invasion, migration, and angiogenesis activity while transfecting miR-221-inhibitor, and AEG-1 siRNA in HCC cells. In addition to that, the upregulation of miR-375 and miR-875-5p markedly induced G1 phase arrest, and the percentage of apoptosis cells increased in the G0 phase. This result confirmed that the overexpression of tumor suppressor miRNAs miR-875-5p [36] and miR-375 [9] promotes cell cycle arrest and apoptosis by the downregulation of AEG-1 in HCC and cervical cancer cells. Our study also shows that knockdown of miR-221 and AEG-1 inhibits cell proliferation, angiogenesis, and induced apoptosis in sub-G0-G1 and G2-M phase also arrested in miR-221 inhibitor or AEG-1 siRNA transfected HCC cells.

The regulation of both the oncomiR and oncogene DNA cluster were studied in glioblastoma cells. Overexpression of miR-26a and CENTG1 promotes cell growth in Glioma cells [37]. In recent years, there have been no studies on the correlation between oncomiR and oncogenes in human cancers, especially miR-221 and AEG-1 in HCC cells. Thus, we focused on both oncogenes regulation in HCC regulatory network. Moreover, we identified the effect of both miR-221 and AEG-1 on their target or associated genes, the regulators of the cell cycle, apoptosis, angiogenesis, and autophagy in HCC cells. The transcription factor LSF/TFCP2 has an oncogenic role and is highly expressed in HCC [38]. Overexpression of LSF transcriptionally upregulates specific genes, such as OPN [39], and MMP9 [40], inducing the level of cell invasion, migration, and angiogenesis activity in HCC cells. In addition to that, LSF identified as a downstream gene of AEG-1 and overexpression of AEG-1 significantly induces LSF mRNA level in HCC cells [41]. On the other hand, OPN regulated by miR-221 and overexpression of miR-221 induces OPN protein levels in osteoblasts [42]. The knockdown of AEG-1 inhibits cell invasion and migration of thyroid cancer cells through the downregulation of MMP2/9 [43]. Besides, overexpression of miR-221/222 inducing the expression level of MMP-9 protein in pancreatic cancer cells [44]. Our results proved that knockdown of AEG-1 and miR-221 significantly downregulates LSF, MMP 9, and OPN expressions in HCC cells.

miR-221 plays a vital role in cell cycle regulation and apoptosis by targeting the regulatory proteins. miR-221 regulates tumor suppressor protein PTEN and suppresses its expression during lung carcinogenesis [45]. The ectopic expression of miR-221 regulates and inhibits the expression of cell cycle regulatory proteins p57 and p27.Inhibition of miR-221 induces cell death by overexpression of p57 and p27 in HCC cells [46]. Another study confirmed that AEG-1 regulates onco-miR mediated tumor suppressor genes such as PTEN, and p57 the target of miR-221 [24]. Our results confirm that knockdown of AEG-1 and miR-221 significantly upregulates these tumor suppressor genes in HCC cells.

The nuclear factor kappa B (NF-κB) is a crucial transcription factor that regulates various pathological and physiological processes, especially cell proliferation, cancer development, and progression. NF-kB is highly activated in cancer cells through the regulation of miRNAs by various mechanisms [47], especially miR-221 [48], and AEG-1 [49]. The activation of canonical and non-canonical (NF-kB) signaling pathway induces the transcription level of Bcl-2 besides, suppressing the PTEN transcription level and promotes cellular functions [50]. Bcl-2 is the direct target of NF-kB and overexpressed the transcription level by the NF-kB transduction pathway in prostate cancer [51]. AEG-1 regulates Bcl-2 protein, and the expression level of Bcl-2 protein was significantly downregulated in AEG-1 siRNA transfected HCC cells [52]. Subsequently, Bcl-2 and BAX proteins regulated by miR-221 and knockdown of miR-221 significantly increased the protein level of BAX and declined Bcl-2 in bladder cancer cells [53]. Furthermore, silencing of PTEN results induced MDM2 mediated p53 degradation through concurrent activation of PI3K/AKT signaling in gastric cancer cells [54].

The overexpression of PTEN modulates tumor suppressor protein RB and inhibits RB phosphorylation by the inhibition of PI-3 Kinase signaling through dephosphorylating the phosphatidylinositol 3,4,5 triphosphate in cervical cancer cells [55]. RB partially regulates NF-kB functions, and pRB suppresses the transcriptional activity of NF-kB in prostate cancer cells [56]. In addition to that, most of the regulatory genes are involved and regulates autophagy function, especially NF-kB [57], PTEN and PI3K/AKT signaling [58], p53 [59], Bcl-2 [60], in a variety of human diseases, including cancer. In this way, the miR-221/AEG-1 axis may regulate LSF, MMP9, OPN, Bcl-2, PI3K, Akt, p57, p53, and RB proteins in HCC. Similar results were obtained in miR-221 inhibitor and AEG-1 siRNA transfected HCC cells.

Hence, based on the previous studies, both miR-221 and AEG-1 involve or regulate multiple cancer pathways, including in HCC. However, whether there is a correlation between miR-221 and AEG-1 in HCC is not yet known. We identified a part of the network, through the association of miR-221/AEG-1 axis in HCC tumorigenesis and both miR-221 and AEG-1 regulate HCC cooperatively.

## 4. Materials and Methods

### 4.1. Cell Lines, Cell Culture

Human HCC cell lines HepG2, Huh7, and Hep3Bwere purchased from National Centre for Cell Science (NCCS), Pune, India was cultured in DMEM with 10% FBS and 1% Penicillin Streptomycin (Invitrogen, Carlsbad, CA, USA). Normal adult liver epithelial cells (THLE-2: ATCC-CRL-2706) were purchased from American Type Culture Collection (ATCC, Manassas, VA, USA), cultured in bronchial epithelial cell growth medium (BMEM) supplemented with 0.08% phosphoethanolamine (Sigma Aldrich Co, St. Louis, MO, USA), 0.06% human recombinant EGF (Corning Inc., Corning, NY, USA) and 10% FBS. Human umbilical endothelial cells (HUVEC) were purchased from Thermo Fisher Scientific (Waltham, MA, USA) and cultured in medium 200 basal media with large vessel endothelial supplement (Gibco). All the cells were cultured in a humidified chamber with 5% CO_2_ at 37 °C.

### 4.2. miRNA and siRNA Transfection

HCC cells were cultured in six-well plates (1 × 10^6^).The transfection was performed after reaching 60% of confluency. miR-221 mimic (4464066), miR-mimic-negative control (HMC0002), miR-221 inhibitor (4464084), miR-Inhibitor-negative control (NCSTUD001) (Thermo Fisher Scientific), small interfering RNA (siRNA) negative control (SIC008), and AEG-1 siRNA (sense: 5′-GACACUGGAGAUGCUAAUAUU-3′, antisense: 5′-UAUUAGCAUCUCCAGUGUCUU-3′) were purchased from Sigma Aldrich, USA and were transfected into the cells with 20 nM concentration using lipofectamine RNAi MAX reagents (Invitrogen) in DMEM medium (serum-free). The mock control cells were treated with transfection reagent alone. The cells were added directly to the transfection complex and replaced with a fresh medium 48 h later. Analysis of the effects of miRNA or siRNA on recipient cells was performed at 48 h after transfection by quantitative real-time-PCR (qRT-PCR).

### 4.3. Quantitative Real-Time PCR

Total RNA was extracted from the RNAi transfected cells using TRIZOL (Invitrogen). For cDNA synthesis, complementary DNA (cDNA) randomly primed from 2 μg of total RNA using the SuperScript IV first-stand synthesis kit (Thermo Fisher Scientific) following the manufacturer’s protocol. qRT-PCR performed by SYBER FAST qPCR master mix (Applied Biosystems) on Step One plus real-time PCR system (Life Technologies, Burlington, ON, Canada). Primers for miR-221, AEG-1, LSF, MMP9, p57, p53, RB, OPN, PTEN, Bcl-2, PI3K, Akt, and LC3A, purchased from Eurofins Genomics India Pvt. Ltd., have been listed in Table S1. U6 snRNA for miR-221 and GAPDH for AEG-1 were used as an internal control. The primer specificity was confirmed by melting curve analysis. Data collected and fold changes of mRNAs and miR-221 were calculated using the 2^−ΔΔ*C*t^ method.

### 4.4. Transwell Migration and Invasion Assay

In the HCC cell invasion assay, the inner surface of the insert coated with Matrigel transwell chamber (2 mg·mL^−1^, BD Biosciences) used, and for the migration assay, the inner surface had no Matrigel-coated transwell chamber used. For transwell invasion assay, cells were transfected with mock control, miR-mimic-negative control, miR-inhibitor-negative control, miR-221 mimic, miR-221 inhibitor, siRNA negative control, and AEG-1 siRNA. After the transfection, cells were collected and seeded (2 × 10^5^) in the upper chamber (8 μm membrane size) containing a serum-free medium. Lower chamber wells were filled with medium containing 10% FBS and incubated for 48 h with CO_2_ at 37 °C. After the incubation, non-invading cells were removed from the upper surface of the filters by wiping with a cotton swab. Invading cells were migrated to the bottom of the membrane and fixed with methanol for 20 min at 37 °C and stained with 0.1% crystal violet. The invasiveness of HCC cells was determined by counting the cells that migrated to the lower side of the filter using a light microscope at 20× magnification (Carl Zeiss, Jena, Germany). For migration assay, the same procedure of invasion assay was performed without Matrigel-coated membrane inserts.

### 4.5. Annexin V-FITC/PI Double Staining of Cell Apoptosis

The Annexin V-FITC/propidium iodide (PI) (V13241, Invitrogen) double staining assay was carried out to detect cell apoptosis on HCC cells. After 48-h transfection, cells were trypsinized, washed twice with PBS, and then resuspended in 100 μL of binding buffer containingannexin mix (5 μL of annexin V-FITC and 1 μL of PI (1 mg/mL)) and left in dark for 15 min at room temperature. After the incubation,an additional 400 μL of the binding buffer was added toeach tube, and the specimens were analyzed within an hour using flow cytometer (BD FACS VERSE (BD, Franklin Lakes, NJ, USA). Flowjo software (version 7.6.5) was used for data analyzing.

### 4.6. Wound-Healing Assay

HepG2, Huh7, and Hep3B cells were seeded in 12 well plates (2.5 × 10^5^) and transfected withmiR-221 mimic, miR-221 inhibitor, AEG-1 siRNA, and their negative controls. After the 90% confluency, the wells were scraped uniformly on the surface of the monolayer using a 200 μL pipette tip. After the wounding, the scraped dimensions were determined and images were captured at 0, 12 h intervals up to 24 h using Floid Cell Imaging Station (Life Technologies, Burlington, ON, Canada). The width of the wound gap was determined using ImageJ analysis.

### 4.7. Propidium Iodide Staining of Cell Cycle Analysis

HCC cells HepG2, Huh7, and Hep3B were collected at 48 h after transfection of RNAi, washed twice with ice-cold PBS and fixed in 70% ice-cold ethanol at −20 °C. After 24-h incubation, they were stained with 250 μL propidium iodide (PI)/RNAs staining solution (50 mg·mL^−1^/1 mg) (MP Biomedicals, Santa Ana, California, USA), and incubated at 4 °C for 30 min dark. Samples were examined using FACS Calibur flow cytometry. Results were analyzed using ModFitLT V3.1 (Beckman Coulter, Porterville, California, USA).

### 4.8. MTT Assay

HCC cells were transfected with miR-221 inhibitor, miR-221 mimic, AEG-1 siRNA, and their corresponding controls. After 48-h transfection, cells were seeded in 96-well plates (1 × 10^4^) and treated with 0.5 mg/mL MTT at 37 °C for 4 h in the CO_2_ incubator. Following the incubation, an equal amount of dissolving solution (0.04 N HCl in isopropyl alcohol) was added to each well and mixed thoroughly to dissolve the crystals of MTT formazan. After the crystals dissolved, the plate read at 540 nm by a microplate reader (Bio-Rad, Hercules, CA, USA). The same procedure was performed at different time intervals (6, 12, and 24 h).

### 4.9. Capillary Tube Formation Assay

One hundred μLof Matrigel matrix (Invitrogen) was added in 24-well plates and left forgel formation overnight at 4 °C. Following gel solidification for 30 min, 50 μLof HUVECs suspension (4 × 10^5^/mL) added to each well. After 48-h transfection of miR-221 inhibitor, miR-221 mimic, AEG-1 siRNA, and their negative controls and the cell culture medium were compensated to 1 mL. The plates were incubated for 16 h at 37 °C. Tube formation was imaged using an inverted microscope (Carl Zeiss). Automated Cellular Analysis System (ACAS) software (version 1.0, 2017-07-14) provided by Ibidi (Munich, Germany) was used to analyze the tube lengths of HUVECs.

### 4.10. Western Blotting Analysis

HCC cells lysate collected from miR-221 mimic, miR-221 inhibitor, AEG-1 siRNA, and their controls transfected HCC cells and were homogenized in RIPA lysis buffer (Santa Cruz Biotechnology, Santa Cruz, CA, USA) after 48 h transfection. Protein concentration was determined using Lowry’s method and total lysate (50 μg per lane) mixed with 4× SDS loading buffer at a ratio of 1:3. Protein samples were heated at 95 °C for 5–7 min and separated on 12% SDS-polyacrylamide gels. The separated proteins were transferred onto a 0.2μm nitrocellulose membrane (Bio-Rad). The membrane was incubated with 5% skimmed milk powder for 1 h in room temperature to block nonspecific antibody binding. After the incubation, the membranes were hybridized with antibodies against AEG-1 (ab124789) (1:10,000), Late SV40 factor (LSF)(ab80445) (1:3000), MMP9 (ab76003, 1:20,000),LC3A/B (ab128025, 1:1000), Osteopontin (OPN) (ab91655, 1:10,000), PTEN (ab32199, 1:10,000), cyclin-dependent kinase inhibitor 1C (p57, Kip2)(ab75974, 1:500), p53 (ab1101, 1:1000), RB(ab24, 1:1000) β–actin (ab6276, 1:5000; Abcam, Cambridge, MA,USA), Bcl-2 (sc-7382, 1:1000), PI3K (sc-1637, 1:1000), and p-Akt (sc-514032, 1:1000, Santa Cruze Biotechnology, Dallas, Texas, USA) overnight at 4 °C. Then, the blots were incubated for 1–2 h at room temperature with alkaline phosphatase (ALP), conjugated anti-rabbit (ab6722), or anti-mouse (ab97020) secondary antibody (1:1000; Abcam, Cambridge, MA, USA). Bands were detected using BCIP/NBT solution (Merk, Millipore, Bedford, MD, USA) and densitometry of Western band was qualified using ImageJ v1.48 software (NIH).

### 4.11. Statistical Analysis

All statistical analyses were performed using Prism software, version 7.0 (Graph Pad Software, La Jolla, CA, USA). The comparison was performed using one-way ANOVA. All the experiments were performed in triplicate and repeated at least three times. *p* < 0.05 was considered statistically significant.

## 5. Conclusions

We showed that miR-221 and AEG-1expressionisupregulated by and associated with HCC tumorigenesis. Recent studies on HCC have shown that oncogenic or tumor suppressor miRNAs and their target gene silencing should be considered for diagnosis and therapy. Our study reveals for the first time how the miR-221/AEG-1 axis is involved in HCC. The expression level of AEG-1 did not alter by miR-221 in HCC cells. On the other hand, the expression level of miR-221 decreased in AEG-1 siRNA transfected HCC cells, and AEG-1 may be associated with miR-221 during RISC formation by optimizing or increasing its activity in HCC. Moreover, the increase in activity of miR-221 leads to the degradation of target/associate genes.

Our study shows that, knockdown of both miR-221 and AEG-1 inhibits cell migration, invasion, proliferation, and angiogenesis, and enhances apoptosis and cell cycle arrest in sub G0-G1/G2-M phases by upregulating PTEN, p57, p53, and RB and downregulating LSF, MMP9, BCL2, PI3K, AKT, and LC3A genes in HCC cells. Furthermore, these findings suggest that the miR-221/AEG-1 axis plays a seminal oncogenic role by modulating PTEN/PI3K/AKT signaling pathway in HCC. Therefore, the miR-221/AEG-1 axis represents a novel therapeutic approach to the treatment of HCC. Nevertheless, the exact direct mechanism of miR-221 and AEG-1 remains unknown during RISC activation. Therefore, further investigations are essential to figure out the relationship between miR-221 and AEG-1 regulation in vivo. In our prospective study, we will further examine the miR-221/AEG-1/RISC axis in NAFLD-associated HCC.

## Figures and Tables

**Figure 1:** Relative mRNA expression levels of miR-221 and AEG-1 in normal liver and HCC cell lines. Relative mRNA expression of miR-221 (**A**) and AEG-1 (**B**) was analyzed in normal liver and HCC cell lines, the expression of miR-221 in miR-221 mimic (**C**) and miR-221inhibitor (**D**) and AEG-1 siRNA (**E**) transfected HCC cells. Relative expression of AEG-1 in miR-221 mimic, miR-221 inhibitor and their control (**F**), AEG-1 siRNA and their controls transfected HCC cells (**G**). All mRNA expressions were performed using qRT-PCR. mRNA expressions were normalized using RNU6 and GAPDH. All reactions were performed in triplicates. Error bars are presented as mean ± s.d. and *** *p* < 0.001, **** *p* < 0.0001. ns: non-significance.

**Figure 2:** miR-221/AEG-1 regulates angiogenesis and cell cycle regulatory mRNA expressions in HCC cell line. Expression level of angiogenesis (LSF and MMP9) and cell cycle (p57, p53, and RB) regulatory mRNAs were analyzed by SYBER Green qRT-PCR in mock control, miR-mimic negative control, miR-inhibitor negative control, miR-221 mimic, miR-221 inhibitor, siRNA negative control, and AEG-1 siRNA transfected HepG2, Huh7, and Hep3B cells using GAPDH as an internal control. Error bars are presented as mean ± s.d. and * *p* < 0.05, ** *p* < 0.01, *** *p* < 0.001 compared with NC group. ns: non-significance.

**Figure 3:** miR-221/AEG-1 regulates apoptosis and autophagy regulatory mRNAs in HCC cell line. The effect of miR-221/AEG-1 on PI3K, Akt, PTEN, OPN, Bcl-2, and LC3A mRNAs expressions analyzed in mock control, miR-mimic negative control, miR-Inhibitor negative control, miR-221 mimic, miR-221 Inhibitor, siRNA-negative control, and AEG-1 siRNA transfected HepG2, Huh7, and Hep3B cells by qRT-PCR using GAPDH as an internal control. Error bars are presented as mean ± s.d. and * *p* < 0.05, ** *p* < 0.01, *** *p* < 0.001, **** *p* < 0.0001 compared with NC control group.

**Figure 4:** Knockdown of miR-221 and AEG-1 inhibits cell migration, proliferation in HCC cells in in vitro. Effect of miR-221/AEG-1 on HCC cell migration and proliferation was analyzed by scratch assay and MTT assay in vitro. HepG2 (**A**), Huh7 (**B**) and Hep3B (**C**) cell lines were transfected with miR-221 mimic, miR-221 Inhibitor, AEG-1 siRNA, and their negative controls. Wound gap distance of cells was quantified in 0, 12, 24 h post-transfection by using Image J (scale bar, 100μm). Cell proliferation was measured by MTT assay in miR-221 mimic, miR-221 inhibitor, AEG-1 siRNA, and their negative control transfected HCC cells (**D**). Error bars are presented as mean ± s.d. and ** *p* < 0.01, *** *p* < 0.001 compared to the negative controls.

**Figure 5:** Downregulation of miR-221/AEG-1 inhibits cell invasion, migration, and angiogenesis in HCC cells. The transwell invasion assay with Matrigel (**A**) and migration assay without Matrigel (**B**) were performed in miR-221 mimic, miR-221 inhibitor, AEG-1 siRNA and their controls transfected HCC cells. Angiogenesis was performed in miR-221 mimic, miR-221 inhibitor, AEG-1 siRNA and their negative control transfected HUVEC cells (**C**). Error bars are presented as mean ± s.d. and ** *p* < 0.01, *** *p* < 0.001 compared to the negative controls (scale bar, 100μm).

**Figure 6:** Inhibition of miR-221 and AEG-1 induces apoptosis and cell cycle arrest in HCC cells. Effect of miR-221 and AEG-1 on apoptosis (**A**) and cell cycle (**B**) was analyzed in mock control, inhibitor negative control, miR-221 mimic, and miR-221 inhibitor, and AEG-1 siRNA transfected HCC cells by flow cytometry. Blue color denotes G2-M phase peak, yellow color denotes S phase peak and green color denotes G0-G1 phase peak; block and red color line denotes sub G0-G1 phase peak. Transfection of miR-221 Inhibitor and AEG-1 siRNA induces apoptosis and cell cycle arrest compared with their negative controls transfected HepG2, Huh7, and Hep3B cells in vitro. Error bars are presented as the mean ± s.d.** *p* < 0.01, *** *p* < 0.001 compared to the control group.

**Figure 7:** Knockdown of miR-221/AEG-1 modulates cell cycle, and angiogenesis regulatory proteins in HCC cell lines. Relative protein expression of AEG-1 in HepG2, Huh7, Hep3B, and THLE-2 cells in vitro (**A**) and in miR-221 mimic, miR-221 Inhibitor, AEG-1 siRNA and their corresponding controls transfected HCC cells (**B**). AEG-1 protein expression level did not alter in miR-221 mimic, miR-221 inhibitor, and their corresponding control transfected HCC cells, and decreased in AEG-1 siRNA transfected HCC cells when compared to their controls. miR-221 and AEG-1 regulatory protein expressions in miR-221 mimic, miR-221 Inhibitor, AEG-1 siRNA and their corresponding controls transfected HCC cells analyzed by Western blot with β-actin used as the internal control. Inhibition of miR-221 and AEG-1 significantly downregulates the expression of LSF, and MMP 9 and significantly upregulates the expression of p57, p53, and RB protein levels in HepG2 (**C**), Huh 7 (**D**), and Hep3B (**E**) cells in vitro. Error bars are presented as the mean ± s.d. and *p*-values are presented as * *p* < 0.05, ** *p* < 0.01,*** *p* < 0.001, **** *p* < 0.0001. ns: non-significant compared to the control group.

**Figure 8:** Knockdown of miR-221/AEG-1 modulates apoptosis and autophagy regulatory proteins level in HCC cell lines. miR-221 and AEG-1 regulatory protein expressions in miR-221 mimic, miR-221 Inhibitor, AEG-1 siRNA, and their corresponding controls transfected HepG2 (**A**), Huh7 (**B**), and Hep3B(**C**) cells analyzed by Western blot with β-actin used as the internal control. Error bars are presented as the mean ± s.d. and *p*-values are presented as * *p* < 0.05, ** *p* < 0.01,*** *p* < 0.001,**** *p* < 0.0001. ns: non-significant compared to the control group.

## Supplementary Materials

Supplementary materials can be found at https://www.mdpi.com/1422-0067/20/22/5526/s1.
